RETRACTED

# Analysis of the Influence of Complexity and Entropy of Odorant on Fractal Dynamics and Entropy of EEG Signal

**DOI:** 10.1155/2016/5469587

**Published:** 2016-09-08

**Authors:** Hamidreza Namazi, Amin Akrami, Sina Nazeri, Vladimir V. Kulish

**Affiliations:** ^1^School of Mechanical and Aerospace Engineering, Nanyang Technological University, Singapore; ^2^School of Metallurgy and Material Engineering, University of Tehran, Tehran, Iran; ^3^Faculty of Cognitive Sciences and Human Development, Universiti Malaysia Sarawak, 94300 Kota Samarahan, Malaysia

## Abstract

An important challenge in brain research is to make out the relation between the features of olfactory stimuli and the electroencephalogram (EEG) signal. Yet, no one has discovered any relation between the structures of olfactory stimuli and the EEG signal. This study investigates the relation between the structures of EEG signal and the olfactory stimulus (odorant). We show that the complexity of the EEG signal is coupled with the molecular complexity of the odorant, where more structurally complex odorant causes less fractal EEG signal. Also, odorant having higher entropy causes the EEG signal to have lower approximate entropy. The method discussed here can be applied and investigated in case of patients with brain diseases as the rehabilitation purpose.

## 1. Introduction

EEG as one of the famous methods for monitoring brain activity specially has been used by scientists in order to study the brain reaction to external stimuli. Scientists have used different approaches to study EEG signals [1–5]. One useful method to study the EEG signal is the fractal method. Fractal time series shows the long-range correlations, meaning that each fluctuation in the time series is correlated with last fluctuations (memory concept), where the correlations change based on power law [6]. Fractal theory has been used widely in biology and medicine in different cases such as DNA [7, 8], human memory [9], bone structure [10], and human stride time series [11].

Olfactory stimulation is one of important types of external stimulation which has aroused the attention of many scientists. Beside the numerous works done on analysis of EEG signal due to olfactory stimulation [12–16], very limited works reported in the literature focus on fractal analysis of the EEG signal in response to olfactory stimuli. In an interesting research Kurihara et al. [17] designed a fractal dimensional map of brain for subjects who received olfactory stimuli. Using this map they studied the activity of different regions of the brain due to stimulation. The result of their analysis showed that cacao or chocolate (as an odor stimulant) had a clearer effect on the fractal dimension of EEG signal compared to the usual fragrant oils. In another research, Murali and Vladimir [18] analyzed the fractal spectra of human EEG signal induced by odors. The result of their analysis showed that fractal approach predicts the EEG signal due to stimulation using different odorants.

RETRACTED

On the other hand, some scientists have analyzed the entropy of EEG signal due to olfactory stimulation. Employing entropy as a measure to analyze the EEG signal due to olfactory stimulation also was very limited. Min et al. [19] computed Shannon entropy of EEG signal as the measure of information content in case of odor stimulation of subjects classified by occupation. Analysis of the averaged entropy from the EEGs of subjects showed that, among the professional perfume researchers, changes of average entropy were more apparent in the frontal region of the brain, while for the general workers and perfume salespersons such changes were more conspicuous in the overall posterior temporal, parietal, and frontal regions. In another work Kroupi et al. [20] used permutation entropy for pleasantness recognition of olfactory stimulus. They showed that the permutation entropy of the EEG conveys olfactory-based information which is able to distinguish between pleasant and unpleasant odors. They also showed that an increase or decrease in the permutation entropy of unpleasant odors with respect to pleasant ones depends on the brain regions. Manzanedo et al. [21] applied three olfactory stimuli on subjects and by analysis of their EEG signal using Shannon entropy. They found out the significant effect of olfactory stimulation on the EEG signal.

Besides all efforts done on analysis of EEG signal due to olfactory stimulation, no study has been reported that relates the complexity and entropy of olfactory stimuli to the fractal dynamics and entropy of EEG signal. In this research we test the complexity and entropy of EEG signal versus the complexity and entropy of odorants, respectively, and show their coupling.

## 2. Method

In order to investigate the effect of odorant's complexity on fractality of EEG signal, the odorant's complexity should be quantified. For this purpose we considered the molecular complexity of odorants. In general, bigger and/or less symmetric molecules have higher molecular complexity. The molecular complexity (*C*) of an odorant is defined using Bertz formula [22]:

(1) $$\begin{array}{c} C=C_{n}+C_{e}. \end{array}$$

In this equation, *C*_*n*_  and *C*_*e*_ are functions of bond connectivity (*n*) and element diversity or kinds of atoms, respectively.

As another parameter to investigate, we study the influence of odorant's entropy at 25°C on the entropy of EEG signal. As it is known, at 0°K odorants have zero entropy and as the temperature increases their entropy increases.

RETRACTED

In order to investigate the influence of odorant's complexity and entropy on fractality and entropy of EEG signal, we selected five pleasant odorants (look at Table 1) from Fenaroli's Handbook of Flavor Ingredients [23].

As it is shown in Table 1, the odorants have molecular complexities in the range of 55.4 (benzyl alcohol) and 177 (diethyl malate). The work by Hendrickson et al. [22] has been used in order to compute the molecular complexities. It was mentioned that, in general, bigger and/or less symmetric molecules have higher molecular complexity.

Also, as it is shown in Table 1, the odorants have entropy in the range of 85.55 (benzyl alcohol) to 145.50 (diethyl malate). The values of odorants' entropies in 25°C were collected from http://realtime.molinstincts.com/.

### 2.1. Data Collection

The experiments were conducted on forty healthy students (20 male and 20 female; 20–22 years old). A physician examined subjects before the experiment to ensure that subjects are healthy. Subjects did not drink beverages which contain alcohol/caffeine within 48 hours before the experiments.

Internal Review Board of the university approved all procedures, and the written informed consent was obtained from subjects, after we explained the study to them.

In order to insulate the subjects, we have done the experiments in an electrically shielded, acoustically isolated, and dimly illuminated room. We instructed the subjects to focus on their breathing while sitting comfortably, without talking and without doing any movement. Also, they were asked to not think about anything.

We diluted odorants in mineral oil in order to equalize their concentrations. We presented each odorant using 10 mL vials. We measured the concentrations of odorants using an olfactometer which was connected to a gas analyzer, to ensure that the resulting vapor concentrations did not differ. The presentation of each odorant to gas analyzer was done 5 times with interstimulus interval of 2 minutes.

The EEG data (with sampling frequency of 256 Hz) were collected using Mindset 24 device. The electrode impedance was kept lower than 5 KΩ. At first, the data collection was done free of any stimulus. Then, we presented different odorants in separate experiments to the subject's nose, and the subject sniffed the odorants, and we recorded the EEG signal. It is noteworthy that we considered interstimulus time of 5 minutes between different odorants' presentations. With the purpose of off-line artifacts rejection, a bipolar EOG was recorded.

RETRACTED

To test the reproducibility of the results, we repeated the data collection where in total two trials were collected from each subject for each stimulus. A physician controlled all experiments.

### 2.2. Data Analysis

Since the recorded EEG data were noisy, first these data were filtered using Wavelet toolbox in MATLAB. After filtering the data, other MATLAB programs computed the fractal dimension and entropy of EEG signals using Box counting [24] and approximate entropy techniques [25].

### 2.3. Statistical Analysis

Mean values of fractal exponent and approximate entropy for the EEG signal were compared between different conditions using one-way repeated measures ANOVA. Mauchly's test (*α* = 0.05) was conducted to test the sphericity. Trend analysis was conducted based on the odorants' properties. Omega squared (*ω* ^2^) was used for a repeated measures design. Effect size, *r*, was employed for pairwise comparisons.

## 3. Results

Here we report the result of analysis. It is noteworthy that all subjects and all trials were included in the analysis. Mauchly's test indicated that the assumption of sphericity had not been violated in case of outcomes (fractal exponent and approximate entropy of EEG signal).

The variations of fractal dimension for EEG signal due to different odorants and the odorants' molecular complexities are shown in Figure 1. The results stand for the mean values.

Since *F*_crit_(5,234) = 2.25 at *α* = 0.05, the result of statistical analysis [*F*(5,234) = 150, *p* = 0.001] stands for the significant influence of odorants on the fractal dimension of EEG signal, with the effect size *ω* ^2^ = 0.69. Generally, odorants reduced the fractality of EEG signal. This result agrees with the result of work reported in [26], which states that the application of stimulus reduces the fractality of EEG signal. Olfactory stimuli conditions had a significant linear trend (*p* = 0.001), indicating that diethyl malate caused a bigger variation in the fractality of EEG signal compared to diethyl succinate, followed by diethyl malonate, dimethyl succinate, and benzyl alcohol, respectively, reflecting the trend of molecular complexity of odorants, that is, diethyl malate bigger than diethyl succinate and bigger than diethyl malonate, dimethyl succinate, and benzyl alcohol, respectively. The effect sizes in Table 2 show that diethyl malate caused the greatest change in the fractality of EEG signal.

The variations of approximate entropy for EEG signal due to different odorants and the odorants' entropy are shown in Figure 2. The results stand for the mean values.

Since *F*_crit_(5,234) = 2.25 at *α* = 0.05, the result of statistical analysis [*F*(5,234) = 69.5, *p* = 0.001] stands for the significant influence of odorants on the entropy of EEG signal, with the effect size *ω* ^2^ = 0.60. Generally, odorants reduced the approximate entropy of EEG signal. This result agrees with the result of work reported in [27], which states that the application of stimulus reduces the approximate entropy of EEG signal. Olfactory stimuli conditions had a significant linear trend (*p* = 0.002), indicating that diethyl malate caused a bigger variation in the approximate entropy of EEG signal compared to diethyl succinate, followed by diethyl malonate, dimethyl succinate, and benzyl alcohol, respectively, reflecting the trend of entropy of the odorants, that is, diethyl malate bigger than diethyl succinate and bigger than diethyl malonate, dimethyl succinate, and benzyl alcohol. The effect sizes in Table 2 show that diethyl malate caused the biggest change in approximate entropy of EEG signal.

RETRACTED

Overall, the coupling between characteristics of odorant and EEG signal was observed, where the odorant having higher complexity and entropy causes the bigger change in fractality and entropy of EEG signal.

## 4. Discussion

In this research we studied the effect of odorant's complexity and entropy on fractality and approximate entropy of EEG signal. Our results demonstrated plasticity of the olfactory-motor phenomenon while smelling different odorants, as the trend of the complexity of odorants is reflected in the trend of the reduction of fractality of EEG signal. For instance, diethyl malate with highest value of molecular complexity caused the biggest variation in EEG signal's fractality, compared to other odorants. This behavior was seen in comparison with other odorants as well. On the other hand, the result of our analysis showed similar trend of variations in case of odorant's entropy and EEG signal's approximate entropy. Overall, the coupling between characteristics of odorant and EEG signal was observed, where the odorant having higher complexity and entropy causes bigger change in fractality and entropy of EEG signal.

The behavior seen in this research can be explained through olfactory perception system. When human smells an odorant, the neurons in the nasal passage send the message to the brain about the odorant which yield to perception [28]. Thus, based on our result, when odorant with higher molecular complexity is sensed by olfactory receptor neurons, these neurons are aroused more and accordingly a stronger message is sent to the brain. Then, this stronger signal has stronger effect on the brain which accordingly is mapped on the EEG signal having lower fractality.

In order to elaborate the behavior seen in variation of approximate entropy we should refer to its definition. Approximate entropy is indicator of randomness of time series where lower value of approximate entropy stands for less randomness. In [6] it was shown that when human receives an external stimulus the EEG signal's Hurst exponent increases from *H* = 0.5 (random state). This increment stands for a less random signal. Thus, here, decreasing the value of the approximate entropy is logical, as by applying the stimulus to subjects, the Hurst exponent increases and accordingly approximate entropy decreases.

RETRACTED

In fact the study done in this research is important due to the method of analysis and the usefulness of its result. Since EEG signal is a chaotic time series that is nonstationary, many of signal analysis methods cannot be used to describe its nonstationary behavior. So, to address the nonstationary behavior of EEG time series, nonlinear processing techniques with their implicit dependence on nonlinear dynamics, chaos, and fractals should be used [29]. As was mentioned before, fractal theory has showed its strength for this purpose as a useful technique.

Entropy also has shown its strength in investigating the dynamics (stochastic rules) of the process generating the trajectory by monitoring the time evolution of the corresponding process. In fact, different types of entropy capture many of the quantitative features of the EEG signal.

On the other hand, rehabilitation has been an important approach in analysis and modeling of neurological signal. Many works investigated the effect of olfactory stimuli on the brains of patients with some neurological disorders [30–33]. In this way, our method of analysis can be investigated for this case to analyze how the odorant's characteristics can affect their brain activity in order to improve its response. Also, our analyses can help the current efforts for the modeling of brain reaction to external stimulation. For instance, the result of our investigation in this research can be linked with our Fractional Diffusion Model brain reaction to external stimulation in [6], in order to write the observed coupling in the mathematical form.

In general, understanding the relation between external stimuli and brain reaction helps the development of the therapy of different brain diseases.

## Figures and Tables

**Figure 1:** Fractal dimension for EEG signal (a) due to different odorants and the odorants' molecular complexities (b). Error bars indicate standard deviations.

**Figure 2:** Approximate entropy for EEG signal (a) due to different odorants and the odorants' entropies (b). Error bars indicate standard deviations.

**Table 1:** Characteristics of odorants.

Name	Compound	Molecular complexity	Entropy (cal/mol·K)
Benzyl alcohol	C_7_H_8_O	55.4	85.55
Dimethyl succinate	C_6_H_10_O_4_	114	118.24
Diethyl malonate	C_7_H_12_O_4_	125	132.42
Diethyl succinate	C_8_H_14_O_4_	135	136.29
Diethyl malate	C_8_H_14_O_5_	177	145.50

RETRACTED

**Table 2:** Effect sizes of pairwise comparisons.

Condition	Fractal dimension effect size (*r*)	Approximate entropy effect size (*r*)
No odorant versus benzyl alcohol	0.59	0.46
No odorant versus dimethyl succinate	0.86	0.78
No odorant versus diethyl malonate	0.91	0.88
No odorant versus diethyl succinate	0.92	0.89
No odorant versus diethyl malate	0.94	0.90
Benzyl alcohol versus dimethyl succinate	0.37	0.33
Benzyl alcohol versus diethyl malonate	0.51	0.52
Benzyl alcohol versus diethyl succinate	0.59	0.59
Benzyl alcohol versus diethyl malate	0.74	0.65
Dimethyl succinate versus diethyl malonate	0.23	0.35
Dimethyl succinate versus diethyl succinate	0.41	0.49
Dimethyl succinate versus diethyl malate	0.70	0.60
Diethyl malonate versus diethyl succinate	0.26	0.26
Diethyl malonate versus diethyl malate	0.67	0.46
Diethyl succinate versus diethyl malate	0.50	0.27
